# 室内空气污染、*HIF*-*1α*基因单核苷酸多态性与福建汉族肺癌易感性的关系

**DOI:** 10.3779/j.issn.1009-3419.2017.03.02

**Published:** 2017-03-20

**Authors:** 斐 何, 琪 祁, 旭 李, 仁栋 肖, 秋萍 徐, 为旻 熊, 志强 刘, 琳 蔡

**Affiliations:** 1 350108 福州，福建医科大学公共卫生学院流行病与卫生统计学系 Department of Epidemiology and Health Statistics, School of Public Health, Fujian Medical University, Fuzhou 350108, China; 2 350108 福州，福建医科大学附属第一医院胸外科 Department of Thoracic Surgery, the First Clinical Medical College of Fujian Medical University, Fuzhou 350108, China

**Keywords:** HIF-1α, rs2057482, 肺肿瘤, 易感性, *HIF*-*1α*, rs2057482, Lung neoplasms, Susceptibility

## Abstract

**背景与目的:**

低氧诱导因子-1α（hypoxia inducible factor 1α, HIF-1α）与肺癌的恶化与转移有关，但*HIF*-*1α*的单核苷酸多态性（single nucleotide polymorphisms, SNPs）与肺癌易感性的研究仍较少。本研究旨在探讨室内空气污染、rs2057482多态性与福建汉族肺癌易感性的关系。

**方法:**

采用以医院为基础的病例对照设计，选择2006年1月-2012年12月在福建医科大学附属第一医院、协和医院和南京军区福州总医院的胸外科及呼吸内科病理确诊的汉族新发原发性肺癌患者1, 096例，选取无肿瘤病史、同期前往医院其他科室探视的患者汉族亲友和社区汉族人群1, 110例，进行问卷调查。应用MALDI-TOF-MS技术对所有研究对象*HIF*-*1α*基因rs2057482位点多态性进行基因分型。

**结果:**

携带有*HIF*-*1α* rs2057482位点T基因型的人群更容易罹患小细胞癌[TT *vs* CC的比值比（odds ratio, OR）值为1.725，95%CI：1.047-2.842s]。调整一般情况和肺癌有关影响因素后，在共显性遗传模型中，暴露于被动吸烟的rs2057482 TT携带者肺癌患病风险是CC携带者的2.195倍（95%CI: 1.038-4.643）。在显性遗传模型中，有肿瘤家族史的rs2057482 T基因携带者肺癌患病风险是C基因携带者的1.911倍（95%CI: 1.121-3.258）。在隐性遗传模型中，肺部疾病史的rs2057482 TT携带者的肺癌患病风险是TC+CC携带者的0.159倍（95%CI: 0.028-0.920）。在加性遗传模型中，有肿瘤家族史的rs2057482 TC+TT携带者的肺癌患病风险是CC携带者的1.542倍（95%CI: 1.107-2.340）。

**结论:**

*HIF*-*1α* rs2057482位点可能与肺癌易感性存在一定关联。

## Abstract (en)

**Background and objective:**

Hypoxia inducible factor-1α (HIF-1α) is associated with the progression and metastasis of lung cancer. There are, however, few studies on the relationship between the single nucleotide polymorphisms of HIF-1α and susceptibility to lung cancer. Therefore, we aimed to investigate the relationship between indoor air pollution, HIF-1α rs2057482, and the susceptibility to primary lung cancer of the Fujian Han population.

**Methods:**

The present study is a hospital-based case-control study. We recruited 1, 096 lung cancer and 1, 110 controls that were admitted to the Department of Thoracic Surgery of the First Affiliated Hospital and Union Hospital of Fujian Medical University and Fuzhou General Hospital of Nanjing Military Region from January 2006 to December 2012. The primary lung cancer cases were identified via pathological methods. Both case and control groups received questionnaires. Genotyping of *HIF*-*1α* gene rs2057482 locus polymorphism in all subjects were analyzed by MALDI-TOF-MS technique.

**Results:**

Individuals who carried the T-genotype of HIF-1α rs2057482 were more susceptible to small cell carcinoma (odds ratio of 1.725, 95%CI: 1.047-2.842). After adjusting for general and lung cancer-related factors, we found that in the co-dominant genetic model, rs2057482 TT carriers were 2.195 times more likely to develop lung cancer than CC carriers (95%CI: 1.038-4.463) in the population that were exposed to passive smoking. In the dominant genetic model, the risk of lung cancer was 1.911 times (95%CI: 1.121-3.258) that in the carriers of the rs2057482 T allele with a family history of cancer. In the recessive genetic model, rs2057482 TT carriers had a 0.159-fold increased risk of lung cancer (95%CI: 0.028-0.920) than TC+CC carriers in people with a history of lung disease. In the additive genetic model, the risk of lung cancer in rs2057482 TC+TT carriers was 1.542 times (95%CI: 1.107-2.340) that in the CC family of people with a family history of cancer.

**Conclusion:**

HIF-1α rs2057482 may be associated with lung cancer susceptibility.

中国是世界肺癌大国，2012年全国数据^[1]^显示每年新发肺癌病例70.5万，发病率36.28/10万人；死亡病例56.9万，死亡率28.81/10万人。肺癌已经连续多年占据中国城市及农村的恶性肿瘤发病和死亡首位。肺部肿瘤生长过程中，血供无法满足肿瘤新生血管供应氧时，肿瘤细胞内即出现缺氧状态，活化低氧诱导因子-1α（hypoxia inducible factor 1α, HIF-1α）识别并结合低氧反应元件（hypoxia response element, HRE）的特殊DNA序列，诱导下游系列靶基因，促进血管生成、细胞增殖及葡萄糖代谢、抑制细胞凋亡、促使肺部肿瘤恶性生长^[2]^。近年来，HIF-1α在肺癌发生发展中的作用逐渐被人们认识，研究^[3, 4]^表明HIF-1α在肺癌组织的表达高于对照组织，并且与肺癌的恶化与转移有关。但*HIF*-*1α*基因单核苷酸多态性（single nucleotide polymorphisms, SNPs）与肺癌易感性的研究仍较少。因此，本研究选择在福建汉族人群中探讨*HIF*-*1α*基因多态性与肺癌易感性的关联，为进一步研究肺癌的发生、发展以及预防和治疗提供一定的科学依据。

## 1 材料与方法

### 1.1 对象

研究对象来自一项持续进行的病例-对照研究^[5]^，选择2006年1月-2012年12月在福建医科大学附属第一医院、协和医院和南京军区福州总医院的胸外科及呼吸内科病理确诊的汉族新发原发性肺癌患者1, 096例，对照组来自同期前往医院探访患者的健康人群和社区健康人群1, 110例，与病例组按性别、年龄（±2岁）进行匹配。所有调查对象均在福建省居住10年以上并且可以清晰回答问题者。研究经过福建医科大学伦理委员会批准，所有面访的调查对象均签署知情同意书。

### 1.2 方法

#### 1.2.1 调查方法

采用统一编制的调查表，由经过统一培训的调查员通过面访形式对所有调查对象进行调查。调查内容包括：一般情况、病例情况、吸烟史、饮酒史、饮茶史、疾病史、职业史、家族史等。应用EpiData 3.1双录入数据，经逻辑纠错，一致性检验，并随机抽样10%复查。吸烟定义为累计吸烟大于100支。环境烟草烟雾暴露按是否在工作场所和/或家庭环境中每日暴露于吸烟者呼出的烟雾时间超过15 min。饮酒定义为每周至少1次，持续半年以上。饮茶定义为每周至少1杯，持续半年以上。装修后有气味定义为装修后入住时调查对象还可以感受到刺激性气味。

#### 1.2.2 实验方法

每例患者与对照抽取外周静脉血5 mL，高速离心分离出白细胞用于提取DNA。应用MALDITOF-MS（美国，Sequenom）技术对所有研究对象*HIF*-*1α*基因rs2057482位点多态性进行基因分型^[5]^。检测结果应用TYPER 4.0软件（Sequenom）完成分型，并输出结果。

#### 1.2.3 统计学方法

采用*χ*^2^检验，比较病例组和对照组在年龄、性别、婚姻状况、文化程度、职业、体重指数（body mass index, BMI）等方面的分布差异，比较病例组和对照组间基因型频率的分布差异；采用非条件*Logistic*回归模型，分析*HIF*-*1α*基因rs2057482位点多态性与肺癌的关联，调整可能的混杂因素后计算调整比值比（odds ratio, OR）值及95%CI；采用分层分析方法评价*HIF*-*1α*基因多态性与肺癌的关联及其与环境因素对肺癌形成的影响；采用*Logistic*回归模型进行相乘模型交互作用的分析；采用相对超危险度比（relative excess risk due to interaction, RERI）、归因比（attributable proportion due to interaction, AP）、交互作用指数（synergy index, S）及其95%CI三个指标估计相加交互作用。统计学检验由SPSS v.23.0软件包完成。所有*P*值基于双侧检验，统计学显著性水平设定为0.05。

## 2 结果

### 2.1 一般情况

截止至2012年12月共收集肺癌病例1, 096例，正常对照1, 110例，病例组的平均年龄为（58.70±10.77）岁，对照组的平均年龄为（59.01±10.83）岁（*t*=0.685, *P*=0.493）；病例组BMI[体重（kg）/身高^2^（m^2^）]为（22.15±3.13）kg/m^2^，对照组为（23.43±3.16）kg/m^2^（*t*=0.468, *P*＜0.001）；其中病例组男性为776例（70.8%）、女性为320例（29.2%），对照组男性为790例（71.2%）、女性为320例（28.8%）。经均衡性检验，发现两组在年龄、性别、婚姻状况方面的分布无统计学差异（*P*＞0.05），但在BMI、文化程度及职业的分布有统计学差异（*P*＜0.05），见表 1。

**1:** 病例组和对照组的一般情况 Demographic characteristics of case and control groups

Characteristics	Demographic characteristics	Case [*n*(%)]	Control [*n*(%)]	*χ*^2^	*P*
		*n*=1, 096	*n*=1, 110		
Gender				0.036	0.849
	Male	776 (70.8)	790 (71.2)		
	Female	320 (28.8)	320 (29.2)		
Education				38.281	＜0.001
	Primary school and below	552 (50.4)	414 (37.3)		
	Middle school	431 (39.3)	549 (49.5)		
	College and above	113 (10.3)	147 (13.2)		
Marital status				2.448	0.118
	Married	1, 034 (94.3)	1, 029 (92.7)		
	Single	62 (5.7)	81 (7.3)		
Occupation				32.458	＜0.001
	Worker	251 (22.9)	281 (25.3)		
	Farmer	277 (25.3)	219 (19.7)		
	Enterprises staffs	267 (24.4)	371 (33.4)		
	Businessman and others	301 (27.5)	239 (21.5)		
Pathological type							
	Adenocarcinoma	519 (47.4)			
	Squamous cell carcinoma	303 (27.6)			
	Small cell carcinoma	90 (8.2)			
	Others^#^	184 (16.8)			
^#^Including adenosquamous carcinoma, alveolar cell carcinoma, large cell carcinoma.					

### 2.2 环境相关因素*Logistic*回归分析

经过性别、年龄、文化程度、职业、婚姻状况及BMI因素调整的*Logistic*回归分析结果提示，室内通风情况不佳（近一年与十年前）、暴露于烹调油烟（近一年与十年前）、吸烟、被动吸烟暴露、饮酒、既往存在肺部疾病史及肿瘤家族史均可不同程度增加罹患肺癌风险，见表 2。

**2:** 肺癌危险因素*Logistic*回归分析 *Logistic* regression analysis of lung cancer risk factors

Variables	Case [*n*(%)]	Control [*n*(%)]	OR (95%CI)	aOR (95%CI)^#^
	*n*=1, 096	*n*=1, 110		
Ventilation				
Well	842 (76.8)	979 (88.2)	1.000 (ref)	1.000 (ref)
Badly	254 (23.2)	131 (11.8)	2.254 (1.791-2.838)^*^	2.283 (1.799-2.896)^*^
Ventilation (10 years ago)				
Well	833 (76.0)	972 (87.6)	1.000 (ref)	1.000 (ref)
Badly	263 (24.0)	138 (12.4)	2.224 (1.774-2.787)^*^	2.321 (1.836-2.934)^*^
Cooking oil fumes				
No	185 (16.9)	344 (31.0)	1.000 (ref)	1.000 (ref)
Yes	911 (83.1)	766 (69.0)	2.211 (1.805-2.709)^*^	2.177 (1.766-2.683)^*^
Cooking oil fumes (10 years ago)				
No	159 (14.5)	274 (24.7)	1.000 (ref)	1.000 (ref)
Yes	937 (85.5)	836 (75.3)	1.931 (1.555-2.398)^*^	1.895 (1.516-2.368)^*^
Decoration				
No	659 (60.1)	685 (61.7)	1.000 (ref)	1.000 (ref)
Odorless	283 (25.8)	288 (25.9)	1.021 (0.840-1.242)	1.054 (0.861-1.291)
Odor	154 (14.1)	137 (12.3)	1.168 (0.907-1.506)	1.254 (0.964-1.631)
Smoking				
No	417 (38.0)	652 (58.7)	1.000 (ref)	1.000 (ref)
Yes	679 (62.0)	458 (41.3)	2.318 (1.954-2.750)^*^	4.175 (3.238-5.383)^*^
Passive smoking				
No	329 (30.0)	616 (55.5)	1.000 (ref)	1.000 (ref)
Yes	767 (70.0)	494 (44.5)	2.907 (2.440-3.464)^*^	2.960 (2.468-3.550)^*^
Alcohol				
No	717 (65.4)	796 (71.7)	1.000 (ref)	1.000 (ref)
Yes	379 (34.6)	314 (28.3)	1.340 (1.119-1.605)^*^	1.337 (1.097-1.631)^*^
Tea				
No	553 (50.5)	534 (48.1)	1.000 (ref)	1.000 (ref)
Yes	543 (49.5)	576 (51.9)	0.910 (0.770-1.076)	0.952 (0.795-1.141)
History of lung disease				
No	960 (87.6)	1, 014 (91.4)	1.000 (ref)	1.000 (ref)
Yes	136 (12.4)	96 (8.6)	1.496 (1.136-1.972)^*^	1.589 (1.191-2.120)^*^
Family history of cancer				
No	882 (80.5)	939 (84.6)	1.000 (ref)	1.000 (ref)
Yes	214 (19.5)	171 (15.4)	1.332 (1.068-1.662)^*^	1.482 (1.178-1.865)^*^
^#^Adjusted by gender, age, educational level, occupation, marital status and body mass index (BMI); ^*^P < 0.05; aOR: adjusted OR.					

### 2.3 rs2057482位点多态性与肺癌易感性的关系

SNP分型结果提示，*HIF*-*1α*基因rs2057482检出率为94.6%。如表 3所示，该位点在1, 110名正常对照中的分布符合*Hardy*-*Weinberg*遗传平衡定律（*P*值为0.05）。说明研究对象具有较好的人群代表性。按照病理类型分类分析的多元*Logistic*回归分析结果显示，携带有*HIF*-*1α*基因rs2057482位点T基因型的人群更容易罹患小细胞癌（TT *vs* CC的OR值为1.725，95%CI：1.047-2.842），尚未发现rs2057482位点多态性与肺癌其他病理类型的关联（表 3）。

**3:** rs2057482与不同病理类型肺癌的易感性关联结果 Association of rs2057482 locus polymorphism with susceptibility to lung cancer of different pathological types

	Adenocarcinoma			Squamous cell carcinoma			Small cell carcinoma			Others			Lung cancer (total)	
	Case/ Control	aOR (95%CI)^#^		Case/ Control	aOR (95%CI)^#^		Case/ Control	aOR (95%CI)^#^		Case/ Control	aOR (95%CI)^#^		Case/ Control	aOR (95%CI)^#^
Co-dominant model														
CC	311/698	1.000 (ref)		193/698	1.000 (ref)		46/698	1.000 (ref)		122/698	1.000 (ref)		672/698	1.000 (ref)
TC	146/304	1.316 (0.764-2.266)		74/304	1.109 (0.556-2.212)		30/304	2.136 (0.773-5.900)		42/304	0.420 (0.126-1.403)		292/304	1.082 (0.871-1.344)
TT	25/48	1.130 (0.872-1.464)		13/48	0.985 (0.709-1.368)		5/48	1.725 (1.047-2.842)		3/48	0.858 (0.581-1.269)		46/48	1.145 (0.716-1.830)
Dominant model														
CC	311/698	1.000 (ref)		193/698	1.000 (ref)		46/698	1.000 (ref)		122/698	1.000 (ref)		672/698	1.000 (ref)
TC+TT	171/352	1.154 (0.903-1.476)		87/352	1.002 (0.734-1.367)		35/352	1.775 (1.101-2.861)		45/352	0.803 (0.549-1.174)		338/352	1.091 (0.887-1.340)
Recessive model														
CC+TC	457/1, 002	1.000 (ref)		267/1, 002	1.000 (ref)		76/1, 002	1.000 (ref)		164/1, 002	1.000 (ref)		964/1, 002	1.000 (ref)
TT	25/48	1.267 (0.740-2.169)		13/48	1.112 (0.561-2.204)		5/48	1.771 (0.654-4.798)		3/48	0.438 (0.132-1.456)		46/48	1.118 (0.702-1.778)
Additive model		1.139 (0.931-1.393)			1.016 (0.787-1.313)			1.584 (1.083-2.316)			0.787 (0.567-1.094)			1.077 (0.908-1.276)
#Adjusted by age, gender, education, BMI, occupation, marital status, ventilation (a year ago), cooking oil fumes (a year ago), decoration, smoking, passive smoking, alcohol, tea, history of lung diseases, family history of cancer.														

### 2.4 环境相关因素分层分析rs2057482位点多态性与肺癌易感性的关系

环境相关因素分层*Logistic*回归分析结果显示：调整一般情况和肺癌有关影响因素后，在共显性遗传模型中，暴露于被动吸烟的rs2057482 TT携带者的肺癌患病风险是CC携带者的2.195倍（95%CI: 1.038-4.643）。在显性遗传模型中，有肿瘤家族史的rs2057482 T基因携带者的肺癌患病风险是C基因携带者的1.911倍（95%CI: 1.121-3.258）。在隐性遗传模型中，有肺部疾病史的rs2057482 TT携带者的肺癌患病风险是TC+CC携带者的0.159倍（95%CI: 0.028-0.920）。在加性遗传模型中，有肿瘤家族史的rs2057482 TC+TT携带者的肺癌患病风险是CC携带者的1.542倍（95%CI: 1.107-2.340）。而在各个遗传模型中，均未见其余因素分层分析时*HIF*-*1α*基因rs2057482位点多态性与肺癌的关联（表 4）。

**4:** rs2057482与肺癌易感性关联的分层分析结果 Stratified analysis of association between four SNPs in rs2057482 and susceptibility to lung cancer aOR (95%CI)^#^

Variables	Stratified	Dominant model	Recessive model	Additive model	Co-dominant model^*^
Gender	Male	1.04 (0.81-1.33)	0.87 (0.50-1.51)	1.00 (0.82-1.23)	1.13 (0.64-1.97)
					1.20 (0.67-2.15)
	Female	1.14 (0.79-1.66)	2.12 (0.85-1.51)	1.21 (0.88-1.65)	0.47 (0.19-1.17)
					0.49 (0.19-1.17)
Ventilation	Badly	1.08 (0.86-1.35)	1.25 (0.75-2.11)	1.09 (0.90-1.31)	0.79 (0.46-1.33)
					0.83 (0.48-1.43)
	Well	1.02 (0.59-1.77)	0.74 (0.26-2.11)	0.96 (0.63-1.47)	1.31 (0.46-3.76)
					1.44 (0.47-4.44)
Cooking oil fume	No	1.10 (0.69-1.76)	1.13 (0.43-2.96)	1.09 (0.75-1.58)	0.86 (0.32-2.27)
					0.94 (0.34-1.44)
	Yes	1.10 (0.87-1.39)	1.17 (0.68-2.01)	1.09 (0.90-1.32)	0.83 (0.48-1.44)
					0.91 (0.51-1.60)
Smoking	No	1.18 (0.88-1.60)	1.13 (0.58-2.19)	1.14 (0.89-1.45)	0.84 (0.43-1.66)
					1.00 (0.49-2.01)
	Yes	0.98 (0.73-1.30)	1.21 (0.61-2.38)	1.01 (0.79-1.28)	0.84 (0.43-1.66)
					0.80 (0.39-1.62)
Passive smoking	No	0.98 (0.71-1.35)	0.64 (0.32-1.29)	0.92 (0.71-1.20)	1.53 (0.76-3.09)
					1.61 (0.78-3.35)
	Yes	1.20 (0.91-1.58)	2.09 (0.99-4.40)	1.24 (0.98-1.56)	1.13 (0.85-1.50)
					2.19 (1.04-4.64)
Alcohol	No	1.10 (0.89-1.37)	1.32 (0.73-2.36)	1.10 (0.90-1.36)	0.74 (0.41-1.34)
					0.79 (0.43-1.46)
	Yes	1.08 (0.74-1.55)	0.86 (0.40-1.85)	1.02 (0.76-1.38)	1.13 (0.52-2.46)
					1.26 (0.56-2.85)
History of lung diseases	No	1.10 (0.89-1.37)	1.39 (0.73-2.36)	1.12 (0.93-1.34)	0.71 (0.43-1.16)
					0.75 (0.45-1.26)
	Yes	0.95 (0.48-1.89)	0.16 (0.03-0.92)	0.73 (0.42-1.29)	1.19 (0.56-2.51)
					0.17 (0.03-1.00)
Family history of cancer	No	0.98 (0.78-1.23)	1.14 (0.67-1.94)	1.00 (0.83-1.21)	0.89 (0.52-1.51)
					0.85 (0.49-1.49)
	Yes	1.91 (1.12-3.26)	1.23 (0.44-3.41)	1.54 (1.02-2.34)	0.65 (0.23-1.83)
					1.30 (0.44-3.86)
^#^Adjusted by age, gender, education, BMI, occupation, marital status, ventilation (a year ago), cooking oil fumes (a year ago), decoration, smoking, passive smoking, alcohol, tea, history of lung diseases, family history of cancer. ^*^In the co-dominant stratification analysis, the first row represents TC *vs* CC, and the second row represents TT *vs* CC. SNP: single nucleotide polymorphism.					

### 2.5 rs2057482位点多态性与环境因素的交互作用分析

根据分层分析结果显示，rs2057482位点显性遗传模型在肿瘤家族史分层分析中存在层间不一致（*P*=0.025），隐性遗传模型在被动吸烟、肺部疾病史分层分析中存在层间不一致（*P*=0.023; *P*=0.020），提示其中可能存在混杂或修饰效应。相乘交互作用分析显示：显性模型下，rs2057482位点多态性与肿瘤家族史之间不存在相乘交互作用（*P*=0.095）。隐性模型下，rs2057482位点与被动吸烟之间存在正相乘交互作用（*P*=0.013），与肺部疾病史存在负相乘作用（*P*=0.016）。进一步分析相加交互作用，结果显示无论是在显性模型还是隐性模型下，rs2057482位点多态性与肿瘤家族史、被动吸烟、肺部疾病史等环境因素之间不存在相加交互作用。

## 3 讨论

空气污染室内空气污染来源多样，烟草烟雾是其重要来源，而装修材料的挥发气体、烹调油烟及居室通风状况等都可能影响室内空气质量，增加肺癌发病风险^[6]^。而室内空气污染则可能降低氧气含量，造成乏氧环境。人类*HIF*-*1α*基因定位于14号染色体（14q21-24），cDNA全长3, 720 bp，编码826个氨基酸^[7]^。当细胞处于乏氧状态时，由于第402位、564位的脯氨酸残基无法被脯氨酰羟化酶（prolylhydroxylase, PHD）所羟化，HIF-1α在细胞内大量积累，并与HIF-1β相结合形成具有转录作用的HIF-1^[8]^。随后，HIF-1可以识别并结合下游靶基因的特定DNA序列，如血管内皮生长因子（vascular endothelial growth factor, VEGF）、促红细胞生成素（erythropoietin, EPO）、诱导型一氧化氮合酶（inducible nitric oxide synthase, iNOS）、血红素加氧酶1（hemeoxygenase-1, HO-1）、糖酵解酶等^[9]^。这些基因的激活可与肺癌的形成、恶化和转移有重要关联^[2]^。尽管*HIF*-*1α*基因的高表达被证实与肺癌的形成与恶化有关^[10]^，但其中的分子机制却仍不清楚，考虑可能与磷脂酰肌醇3-激酶/蛋白激酶B（phosphatidylinositol-3-kinase/protein kinase B, PI3K/Akt）信号通路、细胞因子信号传导抑制蛋白-1、脯氨酸羟化酶PHD家族、基质金属蛋白酶等的反馈调节有关，HIF-1α在肺癌的血管生成、细胞增殖、凋亡、转移、浸润和代谢等中发挥的作用使其有望成为治疗肺癌的一个重要靶点^[11-13]^。到目前为止，关于人类*HIF*-*1α*基因的SNPs有一部分已经被确认，主要有rs11549465、rs11549467和rs2057482。

本研究主要探讨室内空气污染、*HIF*-*1α*基因rs2057482位点多态性与肺癌易感性之间的关联。rs2057482位于*HIF*-*1α*基因3’端非编码区与miRNA-199a的结合区域附近，其多态性可能会影响miRNA-199a的稳定性，从而影响HIF-1α的mRNA和蛋白表达^[14]^。一项与宫颈癌患病风险的研究^[15]^结果显示，携带CC基因型的人群宫颈癌患病风险是携带CT/TT基因型的1.44倍（95%CI: 1.11-1.88）。尽管并未发现*HIF*-*1α*基因rs2057482单个位点与前列腺癌患病风险之间的关联，Li等^[16]^对中国汉族人群*HIF*-*1α*基因多态性和前列腺癌易感性之间的关联研究，通过rs2057482与rs11549467位点结合分析发现，携带≥3个等位基因可使前列腺癌的患病风险增加2.10倍（95%CI: 1.23-3.57）。Qin等^[17]^对该位点与肾细胞癌预后研究，Zhang等^[18]^对该位点与结直肠癌预后研究以及与另一项肝细胞癌预后研究^[19]^结果提示，携带rs2057482 CT/TT基因型的患者较携带CC基因型的患者复发率降低，预后更好。同时发现rs2057482位点多态性可能影响mRNA的稳定性以及和microRNA的结合能力，降低*HIF*-*1α*基因的表达能力和细胞内HIF-1α蛋白的含量，从而产生抗肿瘤效应^[19]^。

本研究结果提示，在全人群中，rs2057482位点T基因型与小细胞肺癌易感性有关联。分层分析结果发现，调整一般情况和肺癌有关影响因素后，rs2057482 T基因携带者在共显性遗传模型中，可增加暴露于被动吸烟人群的肺癌患病风险；在显性遗传模型和加性遗传模型中，可增加有肿瘤家族史人群的肺癌患病风险；在隐性遗传模型中，可降低肺部疾病史人群的肺癌患病风险。Zhang等^[20]^通过培养A549和H157细胞株研究尼古丁与*HIF*-*1α*基因表达的关系，发现尼古丁可通过激活nAchR调节的信号通路来促进HIF-1α蛋白的积累和下游VEGF的表达，对肺癌的形成和恶化起到重要的作用。Guo等^[21]^的研究也得出了类似的结论，研究发现尼古丁可通过诱导线粒体活性氧的产生来调节*HIF*-*1α*基因的表达。因此一定程度上支持本研究结果。而对于危险基因型别的判断，本文结果与Fu、Qin等^[15, 17]^的研究结论不一致，原因可能是研究的肿瘤类别不一致，上述研究种类是肾细胞癌和宫颈癌，不同肿瘤的发病机制不同，故可能会得出不一致的结论，也有可能是研究地区的不同和人群异质性的影响，本研究主要针对福建地区汉族人群rs2057482位点多态性，目前该地区尚无类似的文章可供参考，其他诸如不同的样本量等因素都可能使结论受到影响。

本研究采用病例对照研究设计，样本量较大，将增大结果的可信性；研究针对福建地区的汉族人群，可以排除不同民族人群本身的基因差异对研究结果的影响；研究不仅分析了全人群中*HIF*-*1α*基因rs2057482位点多态性与肺癌易感性的关联，并按照不同病理类型及各类环境因素进行了相应的分类及分层分析，研究了不同亚型人群中rs2057482位点多态性和肺癌易感性的关联，为探讨*HIF*-*1α*基因多态性在肺癌发生发展中的作用机制提供了参考。但研究仍然存在一定的局限：首先以医院为基础的病例对照研究，无法完全排除选择偏倚；其次研究中rs2057482检出率为94.6%，可能与样本质量有关，尽管可能未能成功分型的样本可能会影响结果，但5%左右的未检出率符合质量控制要求，不易造成现有结果方向的改变；本研究仅探讨单基因位点，未能分析基因-基因交互作用，另外未进行功能学研究。因此，未来相关研究可增加检测*HIF*-*1α*基因SNPs的个数或者与肺癌发生有关基因的SNPs（例如DNA修复基因、癌基因和抑癌基因），并在此基础上增加细胞株的培养或采用免疫组化的方法来检测*HIF*-*1α*基因mRNA的水平和HIF-1α蛋白的表达，从而为阐明*HIF*-*1α*基因多态性在肺癌发生发展中的分子机制提供科学的依据，有助于肺癌的预防和后期的临床诊断及治疗，从而提升人群的健康水平。
